# With 3 Types of Respiratory Acquisition: 3.0 T Respiratory Triggered Acquisition Can Obtain Higher Quality DWI Images of the Upper Abdomen

**DOI:** 10.1155/2022/9579145

**Published:** 2022-07-09

**Authors:** Zhuo Shi, Jiuming Jiang, Han Ouyang, Lizhi Xie, Xinming Zhao

**Affiliations:** Department of Imaging Diagnosis, National Cancer Center/National Clinical Research Center for Cancer/Cancer Hospital, Chinese Academy of Medical Sciences and Peking Union Medical College, Beijing 100021, China

## Abstract

**Objective:**

To compare the effects of 1.5 T and 3.0 T upper abdominal magnetic resonance diffusion-weighted imaging (DWI) under three acquisition techniques of breath holding, breath triggering, and free breathing, so as to provide a reference for the usage of upper abdominal DWI scanning.

**Methods:**

Twenty-one healthy subjects were selected from social volunteers and underwent routine magnetic resonance imaging (MRI) and DWI on 1.5 T and 3.0 T, respectively. DWI included three acquisition methods: breath triggering, breath holding, and free breathing, and *b* values were 100 and 800. The DWI image artifacts, image quality, apparent diffusion coefficient (ADC), and the signal-to-noise ratio (SNR) obtained through the three acquisition methods were compared.

**Results:**

The 1.5 T free-breathing DWI image quality was the best, while the 3.0 T had the best breath-triggered DWI image quality. The 3.0 T breath-triggered DWI image quality was better than the 1.5 T free-breathing DWI image (*P*=0.012), and the SNR of free-breathing DWI was the highest. Between the two field intensities, the SNR of the liver in the 3.0 T group was much lower than that in the 1.5 T group, and obvious differences were not observed in ADC values of normal liver, gallbladder, kidney, spleen, and pancreas.

**Conclusion:**

3.0 T respiratory-triggered acquisition can obtain higher quality DWI images. But in the case of only 1.5 T field strength, free-breathing acquisition of DWI images should be selected.

## 1. Introduction

Diffusion-weighted imaging (DWI), which is widely adopted in clinical practice, is a diagnostic technology that uses water molecule diffusion motion characteristics for imaging [1–4]. Without increasing the total scanning time [5], routine MRI sequences have enrolled DWI [6], and currently, DWI is commonly adopted for quantitative and qualitative analyses of organs in the upper abdomen [7]. DWI techniques include respiratory-triggered, breath-holding, and free-breathing acquisitions [4]. The breath-holding technique sacrifices the signal-to-noise ratio (SNR), so the scanning time is relatively short. A higher number of excitations (NEX) is spent by respiratory-triggered DWI under free-breathing status, so images have a high SNR and scanning time is longer [8]. Recently, owing to the rise of DWI with background suppression theory (DWIBS), free-breathing DWI is becoming more and more popular in systemic oncology [9, 10]. In fact, free-breathing DWI can perform thin-layer and multi-NEX scanning, and produce a higher SNR efficiently [11, 12].

Currently, several examinations of the upper abdomen are performed on 3.0 T [13, 14], while a few still operate on 1.5 T in hospitals [15]. However, there are still no available standard scanning regimens or parameters for DWI in the upper abdomen. In the scanning, patients' respiration may vary due to anxiety, tremor, or poor tolerance, which may cause an incorrect apparent diffusion coefficient (ADC) and erroneous diagnosis. Furthermore, artifacts caused by heartbeat and gastrointestinal peristalsis are inevitable, which further decrease the image quality and limit the spreading of DWI applications. Therefore, in our research, images obtained from breath-holding, respiratory-triggered, and free-breathing DWI on 1.5 T and 3.0 T were analyzed quantitatively and qualitatively to select the optimal strategy for upper abdomen DWI clinically.

## 2. Materials and Methods

### 2.1. Subjects

This study is a prospective clinical trial (Registration number: 3332018080). From September to December of 2015, 21 subjects (average age: 47 ± 13 years) were studied, including 13 males and 8 females. The volunteers showed no disease history of organs in the upper abdomen. Exclusion criteria: MRI examination contraindications like implanted pacemaker and claustrophobia. Informed consent was signed by all volunteers, and the experiment was approved by the National Cancer Center/Cancer Hospital, Chinese Academy of Medical Sciences, and Peking Union Medical College ethics committee (Approval number: 21/523–3194). Besides, all experiment steps were performed based on the Declaration of Helsinki.

### 2.2. Methods

On a similar day, an eight-channel body phased-array coil (GE Medical Systems) was adopted to examine volunteers at 1.5 T and 3.0 T scanners (Signa HDxt, GE Medical Systems, Milwaukee, WI, USA). Image collection was conducted through breath-holding, respiratory-triggered, and free-breathing DW-MRI based on single-shot spin-echo echo-planar imaging (SE-EPI), and the *b* values were 100 and 800, respectively. Diffusion direction included frequency encoding, phase encoding, and slice selection. The slice number was 24. The NEX for breath-holding DWI was 1; 2 for respiratory-triggered DWI; and 4 for free-breathing acquisition (Table 1) [16]. The scan range included the whole upper abdomen, and each DWI was scanned 3 times. The data was measured and reported by two seasoned physicians in the Department of Radiology following the blind method, and the GE Z800 workstation was utilized for quantitative and qualitative analyses. The corresponding ADC maps were prepared by the breath-holding, respiratory-triggered, and free-breathing DWI images. Additionally, the ADC value and signal intensity (SI) of the corresponding area were obtained by plotting regions of interest (ROIs) in both DWI and ADC maps. The ROI locations were identical for DWI acquisitions with *b* = 100 and *b* = 800. All the data were measured 3 times, and the mean values represented the final results (Table 1).

### 2.3. SNR and ADC Analysis

The quantitative study included measuring SNR and ADC values. The formula for calculation of SNR was as follows [17]:

(1) $$\begin{array}{c} \text{SNR}=0.655\times \frac{{\text{SI}}_{\text{tissue}}}{{\text{SD}}_{\text{background}}}. \end{array}$$

SI_tissue_ represented the average signal intensity of a certain area and SD_background_ denoted the standard deviation of background measured by selecting the same ROI inside the phase encoding view but outside the tissue (air region of FOV), and SD represented the standard deviation for the signal intensity of the area. Since the background noise in a magnitude image was of Rician distribution rather than the normal distribution, a factor of 0.655 should be added to the SNR calculation. In ADC and DWI maps, the right renal cortex, the right posterior lobe of the liver (main portal vein and its right branch level), the middle portion of the spleen, and the pancreatic tails were the locations of the interested areas.

### 2.4. DWI Artifacts and Image Quality

The images were evaluated by two physicians who were unaware of the study, and image quality was assessed based on artifacts and anatomical structures. Image quality is evaluated using a 4-point scale: Point 1 is very poor, and the image cannot be used for diagnosis; Point 2 is poor, and there are more artifacts that affect the diagnosis; Point 3 is medium, and there are fewer artifacts and the image shows clear anatomical structures; Point 4 is excellent, and the image is clear without artifacts.

### 2.5. Statistical Analysis

The SPSS 24.0 was used to analyze the data. The measurement data were expressed as mean ± standard deviation (SD) and a paired *t*-test was utilized for the comparison. *P* < 0.05 was significantly different.

## 3. Results

### 3.1. Image Quality Comparison of DWI in Three Breathing Modes

The scores of artifacts and image quality remained substantially consistent for the three DWI acquisitions of the upper abdomen (*κ* 0.66∼0.71). As shown in Table 2, the scores of image quality in 1.5 T and 3.0 T for respiratory-triggered, breath-holding, and free-breathing DWI were compared. In three breathing patterns, high *b* values presented more artifacts than low *b* values, and 3.0 T MRI showed higher artifacts than 1.5 T (Figure 1).

Subsequently, we compared the image quality (Table 2). The DWI image quality at *b*_100_ was better than that at *b*_800_ for all three respiratory modes of 1.5 T and 3.0 T. Then, the DWI image quality was compared at *b*_100_ for all three breathing modes: the DWI image quality was best for the 1.5 T free-breathing trigger, while the DWI image quality was best for the 3.0 T breathing trigger, and the DWI image quality was better for the 3.0 T breathing trigger than for the 1.5 T free-breathing trigger (*P*=0.012). These results (Table 2) suggested that *b*_100_ should be selected for examination on 1.5 T with free-breathing acquisition of DWI images, while *b*_100_ should be selected for examination on 3.0 T with respiratory-triggered acquisition of DWI images.

The artifacts with a *b* value of 800 s/mm^2^ showed more number than those with 100 s/mm^2^, and the artifacts of 3.0 T MRI were larger than those of 1.5 T. The lower row *b* = 800 s/mm^2^, and the upper row *b* = 100 s/mm^2^. The right figure was from 3.0 T, and the left figure was from 1.5 T. BH, breath-holding DWI; RT, respiratory-triggered DWI; FB, free-breathing DWI.

### 3.2. Comparison of SNR and ADC of DWI in Three Breathing Modes

As shown in Table 3, irrespective of *b*_100_ or *b*_800_, the SNRs of the kidney, spleen, gall bladder, and pancreas in 1.5 T were lower than those in 3.0 T, while the SNRs of the liver were higher than in 3.0 T and free-breathing DWI exhibited higher SNR of the liver compared with breath-holding and respiratory-triggered DWI (Table 4).

As shown in Table 5, the ADC values of normal organs were not observed with notable differences between the two MRI scanners in normal liver, kidney, gall bladder, pancreas, and spleen when 100 s/mm^2^ and 800 s/mm^2^ were set as *b* values, respectively. Generally, the ADC value of the spleen was the lowest of all the organs. Therefore, different field strengths seemed to have no significant effect on ADC measurement. Among the three acquisition techniques, the mean absolute difference in ADC values between two scans of breath-holding DWI ranged from -0.09 to -0.01 × 10^−3^ mm^2^/s, with consistency limits ranging from ±0.09 × 10^−3^ mm^2^/s to ± 0.48 × 10^−3^ mm^2^/s (Figures 2(a)–2(c)). The mean absolute difference in ADC values between two scans of breath-triggered DWI ranged from −0.04 to 0.01 × 10^−3^ mm^2^/s, with consistency. The limits were between ±0.11 × 10^−3^ mm^2^/s and ±0.17 × 10^−3^ mm^2^/s (Figure 2 D-F). The mean absolute difference between the ADC values of free-breathing DWI between two pairs was −0.07 to -0.02 × 10^−3^ mm^2^/s, and the limits of agreement ranged from ±0.11 × 10^−3^ mm^2^/s to ± 0.18 × 10^−3^ mm^2^/s (Figures 2(g)–2(i)). Considering *b*_800_ of 3.0 T as an example, the worst data of ADC of liver parenchyma in the breath-holding DWI were the 95% confidence interval of the mean difference (limits of agreement) and the mean absolute difference (bias) (Table 6).

## 4. Discussion

Recent studies indicated that there were no statistical differences among breath-holding, respiratory-triggered, and free-breathing DWI in terms of specificity and sensitivity for lesion detection. Furthermore, the image SNR and CNR of free-breathing DWI were the best, with satisfactory linearity between signal intensity (SI) and *b* value, and they had high time efficiency as well [16, 18]. However, the results of this study showed that the best quality of respiratory-triggered DWI images was obtained at 3.0 T field strength and a b-value of 100. However, in the few regions and hospitals where 1.5 T field strength is still used, DWI with a *b* value of 100 and free breathing is recommended [19].

Breath-holding DWI has already been performed in various research projects. Nevertheless, the time the patient holding the breath is a limiting factor for breath-holding DWI, and an increase in the number of diffusion directions, matrix size, number of slices, and number of signal averages is only applicable under certain circumstances. Thus, during breath-holding DWI, the capability of the patient holding the breath should not be exceeded. Conversely, the respiratory-triggered acquisition allows patients to breathe continuously. In this research, an elastic belt was utilized for respiratory triggering. Specifically, respiratory triggering significantly improved signals and provided ADC values similar to breath-holding DWI. Respiratory-triggered DWI can vastly improve image quality, bring higher spatial resolution, achieve multiplanar reformation, utilize multiple and larger *b* values, and then reduce errors in ADC calculation, all with a little time loss. So, respiratory triggering is able to provide patients with much more convenience, especially uncooperative patients. MRI of the liver refers to the approaches about respiratory-triggering modalities [8, 20, 21], with good effects on lesion detection, especially some small lesions [22].

For another thing, respiratory motion is coherent and neither causes any significant mistakes in the ADC measurement nor any obvious decrease in DWI signal [22]. Due to extremely fast single-shot EPI-DWI image acquisition, the images do not suffer from blurring even if patients cannot hold their breath for the entire acquisition. Nevertheless, DW trace images are prepared by fusing single reconstructed images with various motion-probing gradient directions. Despite being of reasonably great quality under free-breathing conditions, these single images (DWIy, DWIx, and DWIs) are not all obtained at an identical stage of respiration. Owing to misalignment between the individuals, the trace-weighted images are not clear enough compared with respiratory-triggered acquisition. So, on account of superior image quality, respiratory-triggered DWI is superior to breath-holding and free-breathing DWI for all the upper abdominal studies, in which the ROIs of organs move with respiration. Improved image quality can also facilitate the detection of lesions, while our study did not address quality questions specifically. Our results showed that when the field strength was 3.0 T, respiratory-triggered DWI had higher image quality and fewer artifacts compared with the other two acquisitions and compared with 1.5 T, the ADC values of normal organs in 3.0 T were stable.

Theoretically, 3.0 T MRI, as the ideal imaging system, can provide two times the SNR compared with 1.5 T and realize the application of high *b* value. Therefore, 3.0 T is more appropriate for the DWI of the upper abdomen [23]. In our study, except for the liver, the kidney, spleen, gall bladder, and pancreas' SNR in 3.0 T was significantly higher than that in 1.5 T MRI. However, geometric distortion due to magnetic susceptibility and signal loss caused by high magnetic sensitivity are challenges associated with 3.0 T [24, 25]. Our study also presented that 3.0 T was more sensitive to motion artifacts compared with 1.5 T, and the images at a high *b* value showed a higher score for artifacts than at a low *b* value. Currently, a few of these issues can be resolved by applying parallel acquisitions or increasing the bandwidth [25, 26].

Theoretically, the ADC value is independent of magnetic field strength, just as shown in this paper. Specifically, though the ADC value of the spleen was lowest among all the epigastrium organs, there was no difference for the liver, gall bladder, spleen, kidney, and pancreas' ADC values between 1.5 T and 3.0 T, and this outcome was consistent with Matsuoka [27] and Notohamiprodjo's [28] reports. By the way, 26 centers (35 MR scanners of 1T, 1.5 T, and 3.0 T) were once involved in a phantom report conducted by Belli et al. [29] The values of the nominal and measured mean ADC in all the centers were observed to be in satisfactory agreement. Over 80% of the mean ADC was within 5% of the nominal value, and 3.5% was the overall standard deviation. Marked differences did not occur in various vendors' ADC evaluations. Chenevert et al. [30] also found that the measured ADC variations of all systems were excellent. Overall, an ice-water phantom or a cylindrical doped water phantom for ADC assessment was identified as the available candidates for application in multicenter tests.

However, our research has certain demerits. For one thing, the sample size was small. All enrolled volunteers were normal, healthy, and cooperative. They differed from patients with diseases in the upper abdomen, whose artifacts and image quality of DWI might vary significantly, and there may be some changes in DWI parameters related to the size of the lesion or pathologies. For another, this report just adopted two *b* values (100 s/mm^2^ and 800 s/mm^2^), and whether the results could be applied to other *b* values still needed more study. Besides, this study lacks the ability to compare with other existing techniques such as navigator-triggered DWI. Though respiratory-triggered DWI is an excellent imaging, some pitfalls, such as irregular breathing patterns or wrongly-placed respiratory belts should be considered. Navigator trigger can resolve these defects. In general, navigator triggering assessing diaphragmatic position with navigator echoes is considered more convenient [31, 32]. In fact, navigator triggering with navigator echoes does not need any external monitoring device, which removes the probability of unexpected interruption of the test caused by respiratory device dislocation. Moreover, this triggering method is not affected by the susceptibility of artifacts because of its additional hardware. Finally, due to variations in parameters among different MRI vendors, generalization of all these conclusions needs to be further investigated.

## 5. Conclusions

To sum up, the image quality of respiratory-triggered DW-MRI on 3.0 T is satisfactory and produces the fewest artifacts. And free-breathing DWI has the highest SNR of the three acquisitions. Although the SNR of most organs in 1.5 T was lower in comparison with that in 3.0 T, the ADC values have no remarkable variation. So, the most appropriate technique for DWI of the upper abdomen is 3.0 T respiratory-triggered acquisition.

## Figures and Tables

**Figure 1:** Images from three different DWIs on 3.0 T and 1.5 T.

**Figure 2:** TheBland–Altman plots of ADC for the normal liver parenchyma in breath-holding (BH), respiratory-triggered (RT), and free-breathing (FB) DWI. ((a)–(c)) The range of consistency limits of ADC values between two scans of breath-holding DWI; ((d)–(f)) the range of consistency limits of ADC values between two scans of respiratory-triggered DWI; ((g)–(i)) the range of consistency limits of ADC values between two scans of free-breathing DWI. The differences of ADC (*y*-axis) were plotted with the mean ADC measurement (*x*-axis) of each two acquisitions; a continuous line represented the mean absolute difference (mean bias), and dashed lines represented the 95% confidence interval of the average difference (limits of agreement). ADC values on the *Y* and *X* axes were ×10^−3 ^mm^2^/s.

**Table 1:** The imaging parameters and techniques of three different DWI on 1.5 T and 3.0 T.

Parameters	Respiratory-triggered (*b*_100_-b_800_)		Breath-holding (*b*_100_-b_800_)		Free-breathing (*b*_100_-b_800_)	
	1.5 T	3.0 T	1.5 T	3.0 T	1.5 T	3.0 T
TR/TE (ms)	6700/75	7500/65	4500/75	4950/65	4500/75	4950/65
Scan time (s)	120	122	23	25	70	72
NEX	2	2	1	1	4	4
Band width (kHz)	250	250	250	250	250	250
Thickness/gap (mm)	5/1	5/1	5/1	5/1	5/1	5/1
Slice	24	24	24	24	24	24
Matrix	128 × 128	128 × 128	128 × 128	128 × 128	128 × 128	128 × 128
Acceleration factor	2	2	2	2	2	2
Diffusion direction	ALL	ALL	ALL	ALL	ALL	ALL
FOV (mm)	360 × 360	360 × 360	360 × 360	360 × 360	360 × 360	360 × 360
Fat suppression	SPIR	SPIR	SPIR	SPIR	SPIR	SPIR

TR, repetition time; FOV, field of view; TE, time of echo; SPIR, spectral presaturation with inversion recovery.

**Table 2:** Comparison of the image quality for three DWI in different field strengths.

B (T)		RT	BH	FB	^1^ *P*	^2^ *P*	^3^ *P*
1.5	b = 100	3.4 ± 0.3	2.6 ± 0.9	3.5 ± 0.4	<0.0001	0.7	<0.0001
	b = 800	2.6 ± 0.6	2.5 ± 0.5	2.8 ± 0.5	0.696	0.3	0.16

3.0	b = 100	4.1 ± 0.2	2.6 ± 0.5	2.2 ± 0.4	<0.0001	<0.0001	0.08
	b = 800	3.2 ± 0.2	2.5 ± 0.4	2.1 ± 0.3	0.003	<0.0001	0.071

BH, breath-holding DWI; RT, respiratory-triggered DWI; FB, free-breathing DWI. ^1^*P*, RT vs. BH; ^2^*P*, RT vs. FB; ^3^*P*, BH vs. FB.

**Table 3:** Comparison of the SNR of different organs in the upper abdomen between 1.5 T and 3.0 T.

	Organ	SNR at *b*_100_			SNR at *b*_800_		
		1.5 T	3.0 T	*P*	1.5 T	3.0 T	*P*
RT	Liver	6.0 ± 1.5	3.7 ± 1.2	<0.0001	3.0 ± 0.7	1.9 ± 0.2	<0.0001
	Gall bladder	41 ± 1.9	60 ± 1.8	<0.0001	4.7 ± 2.6	7.0 ± 2.9	<0.0001
	Kidney	22 ± 2.1	28 ± 2.6	0.001	4.6 ± 1.1	5.5 ± 1.8	0.008
	Spleen	18 ± 9.0	19 ± 2.0	0.401	9.0 ± 3.9	11 ± 7.1	0.002
	Pancreas	9.0 ± 2.9	12 ± 1.9	0.001	3.1 ± 0.6	4.5 ± 1.4	0.001

BH	Liver	4.0 ± 1.0	2.3 ± 0.3	<0.0001	2.2 ± 0.8	1.8 ± 0.9	0.080
	Gall bladder	33 ± 7.0	39 ± 1.8	0.046	2.9 ± 0.3	3.9 ± 1.7	0.002
	Kidney	18 ± 5.9	21 ± 3.0	0.032	3.8 ± 0.6	4.2 ± 0.2	0.141
	Spleen	11 ± 8.0	17 ± 9.0	<0.0001	6.6 ± 4.7	8.0 ± 4.1	0.001
	Pancreas	6.0 ± 1.3	6.6 ± 1.9	0.031	3.0 ± 0.1	3.1 ± 0.8	0.902

FB	Liver	6.9 ± 3.0	5.8 ± 2.1	0.003	3.5 ± 0.7	2.4 ± 1.0	0.004
	Gall bladder	56 ± 9.0	61 ± 1.7	0.015	9.0 ± 2.9	11 ± 5.0	0.002
	Kidney	29 ± 3.9	36 ± 1.1	0.001	6.1 ± 1.8	6.9 ± 3.0	0.024
	Spleen	23 ± 1.9	26 ± 1.6	0.081	11 ± 4.9	12 ± 8.9	0.217
	Pancreas	12 ± 7.0	15 ± 7.0	0.001	6.0 ± 1.0	7.0 ± 2.0	0.011

RT, respiratory-triggered DWI; SNR, signal-to-noise ratio; FB, free-breathing DWI; BH, breath-holding DWI.

**Table 4:** Comparison of the liver SNR of the three DWIs in 1.5 T and 3.0 T.

(T)	b	RT	BH	FB	^*1*^ *P*	^*2*^ *P*	^*3*^ *P*
1.5	*b* = 100	6.0 ± 1.5	4.0 ± 1.0	6.9 ± 3.0	0.001	0.006	<0.0001
	*b* = 800	3.0 ± 0.7	2.2 ± 0.8	3.5 ± 0.7	0.002	0.005	0.001
3.0	*b* = 100	3.7 ± 1.2	2.3 ± 0.3	5.8 ± 2.1	0.001	<0.0001	<0.0001
	*b* = 800	1.9 ± 0.2	1.8 ± 0.9	2.4 ± 1.0	0.6	0.016	0.012

BH, breath-holding DWI; RT, respiratory-triggered DWI; FB, free-breathing DWI.

**Table 5:** The ADC of normal organs in the upper abdomen between two field strengths with *b* values as 100 s/mm^2^ and 800 s/mm^2^.

Organs	*b* = 100			*b* = 800		
	1.5 T	3.0 T	*P*	1.5 T	3.0 T	*P*
Liver	2.8 ± 0.51	2.8 ± 0.34	0.41	1.2 ± 0.14	1.1 ± 0.37	0.27
Gall bladder	3.6 ± 0.70	3.6 ± 0.85	0.53	2.4 ± 0.40	2.4 ± 0.30	0.91
Kidney	3.4 ± 0.72	3.4 ± 0.61	0.57	1.7 ± 0.10	1.6 ± 0.90	0.32
Spleen	1.2 ± 0.23	1.2 ± 0.25	0.86	0.69 ± 0.030	0.67 ± 0.10	0.28
Pancreas	3.2 ± 0.74	3.2 ± 0.63	0.58	1.1 ± 0.35	1.1 ± 0.24	0.51

The unit of ADC value is *mm*^*2*^*/s*.

**Table 6:** The mean absolute difference (bias) and 95% confidence interval of the mean difference (limits of agreement) of ADC of liver parenchyma from the three DWIs.

DWI	Series of scans	Mean bias	Limits of agreement
Respiratory-triggered	1 vs. 2	−0.04	±0.11
	1 vs. 3	−0.03	±0.15
	2 vs. 3	0.01	±0.17

Breath-holding	1 vs. 2	−0.01	±0.09
	1 vs. 3	−0.09	±0.48
	2 vs. 3	−0.08	±0.47

Free-breathing	1 vs. 2	−0.02	±0.11
	1 vs. 3	−0.07	±0.14
	2 vs. 3	−0.06	±0.18

## Data Availability

The data used to support the findings of this study are available from the corresponding author upon request.

## Abbreviations

DWI: Diffusion-weighted imaging
MRI: Magnetic resonance imaging
ADC: Apparent diffusion coefficient
SNR: Signal-to-noise ratio
NEX: Number of excitations
SE-EPI: Spin-echo echo-planar imaging
SI: Signal intensity
ROIs: Regions of interest
RT: Respiratory Triggered
BH: Breath-holding
FB: Free breathing
TR: Repetition time
FOV: Field of view
TE: Time of echo
SPIR: Spectral presaturation with inversion recovery.
